RETRACTED

# An Intelligent Classification System for Cancer Detection Based on DNA Methylation Using ML and Semantic Knowledge in Healthcare

**DOI:** 10.1155/2022/4334852

**Published:** 2022-10-10

**Authors:** Anuradha Thakare, Manisha Bhende, Mulugeta Tesema, Mohammed Dighriri, R. Bhavani, Amena Mahmoud

**Affiliations:** ^1^Department of Computer Engineering, Pimpri Chinchwad College of Engineering, Pune, India; ^2^Marathwada Mitra Mandal's Institute of Technology, Pune, India; ^3^Department of Chemistry (Analytical), College of Natural and Computational Sciences, Dambi Dollo University, Dambi Dollo, Oromia Region, Ethiopia; ^4^Department of Basic Sciences and General Requirements -IT skills, Fakeeh College for Medical Sciences (FCMS), Jeddah, Saudi Arabia; ^5^Department of CSE, Saveetha School of Engineering, Saveetha Institute of Medical and Technical Sciences, Chennai 602105, India; ^6^Computer Science Department, Faculty of Computers and Information, Kafrelsheikh University, Kafr El Sheikh, Egypt

## Abstract

To consistently assess a patient's internal and external wellness and diagnose chronic conditions like cancer, Alzheimer's disease, and cardiovascular disease, wearable sensing devices are being used. Wearable technologies and networking websites have become incredibly common in the medical sector in recent times. The condition of a patient's health can be influenced by a number of factors, including psychological response, emotional stability, and anxiety levels, which can be evaluated using social network analysis based on graph theory-based techniques and these ideas, known as “social network analysis” (SNA) are used to study relationship phenomena. Therefore, numerous uses for SNA in health research are possible, ranging from social science to exact science. For example, it can be used to research cooperative networks of healthcare providers and hazard-prone behaviors, infectious disease transmission, and the spread of initiatives for health promotion and prevention. Recently, a number of machine learning-based healthcare solutions have been proposed to track chronic illnesses utilizing data from social networks and wearable monitoring devices. In our suggested approach, we are using an intelligent system with the assistance of wearable sensors for the classification of cancer based on DNA methylation, an important epigenetic process in the human genome that controls gene expression and has been connected to a number of health issues. A mixed-sampling imbalanced data ensemble classification technique is created with the help of biomedical sensors to address the problem of class imbalance and high dimensionality in the Cancer Genome Atlas (TCGA) massive data. This technique is based on the Intelligent Synthetic Minority Oversampling (SMOTE) algorithm. The false-negative rate significantly rises as a result of this, to give a larger data set, a new minority class sample will be first obtained. The noise created during the sample expansion process is actually any data that has been acquired, preserved, or altered in a way that prevents the system that initially conceived it from accessing or utilizing it. Noisy data boosts the amount of space needed excessively and can also drastically influence the findings of any data collection investigation and therefore can also affect the sample sets of one or the other class, resulting in the class imbalance which acts as a common problem in ML datasets. The Tomek Link method is then used to eliminate this noise, producing a reasonably balanced data set. Each layer selects two random forest structures using the cascading forest structure of the deep forest (GC-Forest) algorithm to increase the generalization ability of the model and create the final classification model. Experiments using DNA methylation data collected by employing biosensors from six tumor patients reveal that the mixed-sampling unbalanced data ensemble classification technique may increase the sensitivity to the minority class while maintaining the majority class's classification accuracy.

RETRACTED

## 1. Introduction

The manufacturing of therapeutic devices has advanced much in the last 20 years, with attention to the significance of sustaining human health. Biomedical sensors are being utilized more extensively as wearable devices that enable real information monitoring, such as fitness trackers, wristbands, and watches. Possessing smart materials integrated into them that track real-time data (heart rate, blood glucose, plasma levels, etc.) to guide healthcare professionals. As promising tools for online human research, devices have thus been in surge demand. Current method followed cancer monitoring and other diseases that ought to be attached to critical ports for machine learning and deep forest approach neural networks for ailment detection. In recent years, predictive models of cancer classification combined with biological and genetic data have enabled a more accurate assessment of cancer risk [1]. DNA methylation has become one of the most important epigenetic modifications in cancer research, with studies showing abnormal DNA methylation patterns in “tumor” tissues compared to “normal” tissues [2]. Using machine learning (ML), massive and difficult data sets can be incorporated. The patient experience and outcomes might be optimized by employing these data sets. The creation of functional genomic is tightly linked to a specific treatment approach. Genetic code collection, for instance, may rise by double factors every two years. In contrast, the speed of innovation in a virtual machine has been exceeded by the rise in computational power, linked with the quick reduction in the expense of genotyping. Thus it is only happening with the miracles of ML. Therefore, a new line of research in the field of biological information involves applying machine learning theories and techniques to locate oncogene-related DNA methylation regulatory sites, examine the mechanisms behind the development and incidence of cancer, and discover fresh cancer indicators [3].

RETRACTED

The Cancer Genome Atlas (TCGA) is currently one of the most comprehensive cancer sequencing databases, and the rich cancer sample data provides a prospect for developing cancer classification models [4]. The TCGA is a research that employs genetic sequencing and bioinformatics to assemble a list of genetic alterations that cause cancer and thereby plays a significant role in DNA sequencing. The key aim was to implement increased DNA sequencing approaches to improve the diagnosis of cancer, management, and control through a profound understanding of the genomics of the ailment. Like most data, the data in TCGA is inherently imbalanced, which means one or more classes have significantly lower proportions in the training data than the other classes. There is an imbalance resulting in the wrong classification in the detection and identification of cancer sequencing, and this issue can also be termed as the high dimensional and class imbalance data. The classification of these highly imbalanced data suffers from the majority class, resulting in increased false negative rates [5]. A mixed-sampling imbalanced data ensemble classification technique based on the Intelligent Synthetic Minority Oversampling (SMOTE) algorithm is developed with the help of biomedical sensors to address the problem of class imbalance and high dimensionality in The Cancer Genome Atlas (TCGA) massive data.

Hence, to solve the problems of class imbalance and high dimensionality issues in the data set of cancer classification model, the main contribution of our study is to propose an integrated intelligent classification model embedded with biomedical sensors and mixed sampling. The minority sample set is expanded using the intelligent SMOTE method, and the boundary and noise data are removed using the Tomek Link algorithm, resulting in generally balanced training data. On the basis of ensuring the classification accuracy of the majority class, it also imports the training data into the Gcforest model and successfully improves the classification accuracy of cancer minority class samples.

RETRACTED

The ML and DL techniques employed in the analysis of cancer development are explored in this work. The bulk of predictions mentioned is associated with particular ML inputs and targeted sample management [6]. To improve academic approaches and prepare the way for information and analyse of medical research, we focused on analyzing and evaluating countless research AI and machine learning approaches, strategies, and perspectives in this study [7]. To categorize the various cancer kinds according to the tissue from which they emerged, we employed SVM, Naive-Bayes, Extreme-gradient-boosting, and RF machine learning models. RF outperformed the other predictors, achieving 99% reliability. In fact, we employed local interpretable model-agnostic explanations to assess relevant methylated patterns to identify specific disease classifications [8]. The vision of medical guidance will move toward speedier modeling of a new medication for each patient via medical application of machine learning and artificial intelligence in cancer diagnosis and therapy. Experts may work together in real-time and disseminate expertise digitally using the AI-based systematic approach, which has the power to heal millions of citizens. By fusing genetics and intelligent systems, the study presented game-changing medical innovations in this study and highlighted how oncologists might gain from intelligence support for focused cancer care [9].

### 1.1. Organization

The study is organized into several modules where the first module provides the introduction to the problem statement followed by the 2^nd^ section which states about the various methods involved in the study.  Section 3^rd^ discusses about the analysis and discussions regarding the experiments conducted and investigations performed, followed by the ultimate section which provides the conclusion of the study.

## 2. Methods

The mehods here, are separated into three stages: data preparation, feature selection, and model training and validation. In the preprocessing step, the intelligent SMOTE algorithm is employed to maintain a balanced class distribution, and the Tomek Link under-sampling approach is utilized to remove noise from the data which is the main parameter that is considered in the gene sequencing because noisy data boosts the amount of space needed excessively and can also drastically influence the findings of any data collection investigation, therefore, affects the sample sets of one or the other class resulting in the class imbalance which acts as a common problem in ML datasets. Thus, only genes with cancer-causing mutations were examined to limit the data's feature space. COSMIC and CIVic Internet database resources were used to collect data. Create a classification model using the Gcforest technique, the model was tested on six distinct forms of cancer obtained from biomedical sensors embedded on the patient's body [6, 10]. The data on DNA methylation came from https://portal.gdc.cancer.gov/repository.  Figure 1 displays the technical flow chart of the research in this paper.

RETRACTED

### 2.1. Data Preprocessing

#### 2.1.1. Data Processing

DNA methylation data for 28 cancer types was released by the TCGA study. Raw data (0 × 1) may be downloaded from the TCGA website and mapped to particular data spots or ranges (eg, chr19 : 19033575 indicates location 19033575 on chromosome 19). The Broad Institute's FireBrowse, which maps numerical values to particular human genes labelled using HGNC nomenclature, is used to preprocess DNA methylation data in this research [7, 8]. Each sample file has a TCGA identification number that specifies whether it is a tumor tissue or a normal tissue (e.g., TCGA-2F-A9KW-01: tumor type: 0109 (category 1), normal type: 10 19). (Category 0) [9].  Table 1 shows the statistics of six tumor types from the TCGA database that has quite extensive sample data.

#### 2.1.2. Sampling

The data from TCGA is substantially skewed, as seen in Table 1, due to the nonuniform distribution of the target classes. For cancer samples, current classification algorithms offer good accuracy, but limited sensitivity for normal samples [11]. As a result, this research provides a mixed sampling approach that is used when a sample strategy calls for the use of two or more fundamental sampling techniques. These approaches are employed for evaluating and modifying processes that influence the execution of evidence-based solutions. These techniques further optimizing the normal sample sensitivity while maintaining excellent accuracy.

*(1) Technique of Intelligent Synthetic Minority Sampling (ISMOTE)*. The author has presented Intelligent SMOTE (Intelligent Synthetic Minority Oversampling Technique), an enhanced approach based on the random oversampling algorithm [12]. To balance the dataset, fresh samples are inserted into a limited number of comparable samples. Rather than using a random oversampling approach that just copies the sample, the SMOTE algorithm creates a fresh sample from scratch, bypassing some categorization filtering. The SMOTE algorithm works on the following principle:

(1) Calculate the distance between each sample *x* in the minority class and all samples in the minority class sample set using the Euclidean distance as the standard, and determine its *k* closest neighbors.
(2) Determine the sampling ratio N based on the sample imbalance ratio, then randomly choose multiple samples from the k-nearest neighbors for each minority class sample *x*.
(3) Create a new sample from the old sample using the procedure for each randomly picked neighbor (1).
  (1) $$\begin{array}{c} p_{i}=x+rand\left(0,1\right)\times \left(y_{i}-x\right),i=1,2,\ldots \ldots ,N\text{,} \end{array}$$
where *x* is the sample, rand (0,1) represents a random number in the interval (0,1), and *y*_*i*_ is the *k*-nearest neighbors.

*(2) Tomek Link*. The concern is that while the Intelligent SMOTE approach extends the sample space of the minority class while balancing the class distribution, the space initially belonging to the majority class sample may be “invaded” by the minority class, resulting in model overfitting. To overcome this issue, the Tomek Link method [13] is used to remove noise points or boundary points, which effectively solves the “intrusion” problem. The Tomek Link algorithm is based on the following principle: assume that the sample points *x*_*i*_ and *x*_*j*_ belong to separate categories, and that the distance between them is represented by *d*(*x*_*i*_, *x*_*j*_). If there is no third sample point xl such that *d*(*x*_l_, *x*_*i*_) < *d*(*x*_*i*_, *x*_*j*_) or *d*(*x*_*l*_, *x*_*j*_) < *d*(*x*_*i*_, *x*_*j*_) holds, call (*x*_*i*_, *x*_*j*_) a Tomek Link pair. If two sample points are Tomek Link pairs, one of the samples is either noise (too much deviation from the normal distribution) or both samples are on the border between the two classes. It means that these assumptions are necessary to make separate categories of the data to analyse the noise and the normal data set. These assumptions are mandatory for the removal of ambiguity. Furthermore, by inserting the Euclidean distance between the sample point and the original sample point and its neighbors, the research in this article ensures that the inserted data has a fair resemblance with the original sample. The Tomek Link technique is employed after the SMOTE algorithm has extended the minority samples. The Euclidean distance is calculated and sample points with low similarity, referred to as noise points or boundary points in the text, are discarded.

RETRACTED

#### 2.1.3. Blood Pressure Measurement Using Biomedical Sensors

Blood pressure is one of the four vital signs of the human body, which can reflect the systolic function of the heart. The pulse transit time (PTT) is the core principle of noncontact blood pressure measurement. It was initially estimated by ECG and PPG jointly, and then the author measured it by two rPPG signals, which opened the rPPG noncontact measurement of blood pressure prelude. From the literature, the calculation formula of BP estimated by PTT can be known as follows:

(2) $$\begin{array}{c} BP=b+c*PTT\text{.} \end{array}$$

*B*, *c* are related to the elasticity of human blood vessel walls. Based on this concept, the author proved for the first time that the value of multipoint PTT of the body can be calculated in a noncontact way and developed a noncontact multiparameter measurement system based on this. The author has designed a framework for adaptively selecting rPPG modules based on the Gaussian model and proved the high correlation between PTT and BP by analyzing the characteristics between rPPG signals [13]. The quality of the signal pulse plays a vital role in estimating PTT based on rPPG. Authors improved the Kalman filter to improve the signal-to-noise ratio of the rPPG signal and show more apparent peaks to improve the estimation accuracy of PPT. In addition, the blood pressure monitoring method based on multipoint pulse wave phase difference has also been proved to have good measurement accuracy in addition to the PTT estimated by the single-point signal peak due to the influence of the body's voluntary movement. The author collects signals from the radial artery of the left hand and the end of the finger to calculate the PPT. The experiment proves that the correlation between the calculated PTT and blood pressure reaches 0.79, which is higher than that of the single-point pulse wave phase difference calculation method that only uses a single signal to calculate the PTT. However, the author also pointed out that the multipoint measurement method has higher requirements on the camera's frame rate.

#### 2.1.4. Heart Rate Variability Measurement Using Biomedical Sensor

HRV, a parameter closely related to heart disease, is an essential indicator of whether the heart rate is abnormal. ECG has always been the standard equipment for HRV detection, and the characteristics of QRS complexes analyse the difference between heartbeat cycles in terms of clinical use. Studies have shown that the pulse wave and HRV signal have an equivalent relationship. Still, the time-domain parts of rPPG movement are easily affected by noise, and pulse wave signal characteristics (64) have become an effective method. Each skin patch provides a pulse signal, which is selected from the time domain and frequency domain features of multiple passwords and combined with practical information to improve the discriminability of rPPG for abnormal heart rate detection under noise and unnatural interference. In addition, atria fibrillation can lead to abnormal PPG signals. Therefore, Pereira et al. proposed a dual-window support vector machine classification model based on this feature. After testing, the model showed good performance on a dataset consisting of many patients. Generalization performance and test performance; also using the dual-window detection strategy, authors used the periodic variance maximization algorithm to extract the rPPG signal. Periodic Variance Maximization also is a newly developed technique used to extract the cardiac signal embedded within the RGB temporal patterns in remote-photo-plethysmography-signal (rPPG). By integrating the two strategies, the PVM algorithm seeks to determine the required signal's unknown period. Two procedures are used: first, an incremental subdomain dissection process that creates a periodicity-maximizing basis for a particular frequency, then secondly, a global optimization tabu search algorithm is employed to identify the frequency with the highest global periodicity across the search space. For any type of biosensor measuring scenarios without vibration, the suggested technique is utilized to retrieve any desired signal of deviations from a blend of data and can adaptively detect the peak through the dual-window, which successfully improved the detection effect of rPPG on HRV. In the frequency domain, the power information of high frequency and low frequency is another indicator of whether the heart rate information is abnormal. Still, it is also easily affected by noise. The author separated the noise and signal into independent components based on ICA, showing better experimental results than EVM. HRV analysis based on rPPG is still in the laboratory stage, and the clinical use, and diagnosis of other arrhythmia-related physiological diseases based on HRV will be the focus of future research.

RETRACTED

### 2.2. Data Preprocessing

The TCGA DNA methylation data in diverse cancer types include about 20 000 protein-coding genes as distinctive characteristics. Feature selection is critical in this instance [14]. As a result, only those genes that have been scientifically recognized as having cancer mutational importance are targeted by the research. The Cancer Gene Census (COSMIC) and Clinical Interpretation of Variants in Cancer (CIVC) were used to find these genes (CIVic). The COSMIC Cancer Gene Census (CGC) is a benchmark in cancer genetics used in fundamental research, medical reporting, and pharmaceutical development. It is an elite description of the genomes creating human cancer. While as (CIVic) describes the therapeutic, predictive, analytical, and inducing relevance of hereditary and physiological variations of all types. CIVic is an elite aspect of learning for Clinical-Interpretation-Variants in cancer. To facilitate the transparency and open generation of current and reliable variant analyses for use in cancer targeted therapies, CIVic is dedicated to accessible code, increased samples, accessible app programming interfaces (APIs), and traceability of substantiating evidence.

RETRACTED

### 2.3. Intelligent Classification Model

Authors devised the Gcforest technique, a decision tree-based ensemble algorithm [15]. The two essential elements that make up the core of Gcforest are Cascade Forest and MultiGrained Scanning. The makeup of the Cascade Forest is as follows: The decision trees that make up each forest in the cascade forest are composed of a number of random and utterly random forests. Random forests at each layer and overall ensure the model's heterogeneity.  Figure 2 depicts the particular cascade forest structure.

Two full random forests (black) and two random forests (red) make up each layer of the cascade forest in Figure 3 (blue). Each random forest also contains 30 entirely random decision trees, each of which randomly chooses a feature for splitting until the examples contained in each leaf node belong to the same class. The best base value for splitting is picked for each decision tree by selecting sqrt (*d*) features (the sum of the features of *d* inputs) at random. When the effect cannot be further enhanced, the cascade forest iteration comes to an end.

Each forest contains many decision trees, each of which will determine a class vector result (for example, three classes, as shown below), then combine all decision tree results, and then take the mean to generate the forest's results. The final decision result is a three-dimensional class vector, and Figure 4 depicts the decision process for each forest. Each forest will choose a three-dimensional class vector in this manner. Returning to Figure 3, each of the four forests in the cascade forest can choose a three-dimensional class vector, then average the four class vectors, and finally take the highest value. The final classification result is the category that corresponds to the value.

### 2.4. Evaluation Indicators

Recall/Sensitivity-: The larger the value of Sen/Rec, the larger the disease is judged to be diseased, and the smaller the missed detection (FN).

(3) $$\begin{array}{c} Rec=Sen=\frac{TruePositive}{TruePositive+FalseNegative}\text{.} \end{array}$$

Precision-: Precision, that is, the proportion of all positive predictions that are correctly predicted.

(4) $$\begin{array}{c} Prec=\frac{TruePositive}{TruePositive+FalseNegative}\text{.} \end{array}$$

*F*_1_ is the ratio of the arithmetic mean to the geometric mean, the bigger the better.

(5) $$\begin{array}{c} F_{1}=2\times \frac{Prec\times Rec}{Prec+Rec}\text{.} \end{array}$$

The response sensitivity and specificity ROC curve is a comprehensive measure of continuous variables. It allows for a natural comparison of various trials on the same scale. The bigger the diagnostic value, the more convex and closer the ROC curve is to the top left corner, which is useful for comparing various indicators the area under the curve may be used to assess the diagnostic accuracy.

RETRACTED

## 3. Analysis and Discussion

Training set: test set ratio of the DNA methylation data using biomedical sensor received from TCGA is 7 : 3.  Figure 5 illustrates the PCA 2D plot of the training data, which demonstrates that the sample data distribution is extremely imbalanced.

Table 2 shows the model performance comparison of four classification methods, CcForest, Logistic Regression (LR), Random Forest (RF), and Deep Belief Network (DBN), and the same indicators has been represented in Figure 6 [16, 17]. It can be seen from Table 2 that the four classification algorithms have high accuracy for the majority class samples, but poor sensitivity on the minority class, which is caused by the imbalance within the data [18].

To solve the above problems, the SMOTE algorithm proposed in this paper is combined with the mixed sampling model of the TomekLink algorithm to preprocess the DNA methylation data. The PCA two-dimensional map of the processed DNA methylation data is shown in Figure 7, and the data distribution is relatively balanced [19].

After the data obtained from bio medical sensors are standardized, the four classification models are compared again. As shown in Table 3, after using the mixed sampling model proposed in this paper, the evaluation indicators Sen/Rec, Pre, and *F*_1_ of the four classification models for the minority class have been greatly improved.

Comparing Table 2 and Table 3, it can also be found that among the four classification models and Figure 8 demonstrates the performance indicators of the four models after mixed sampling, whether before or after sampling, the Gcforest algorithm has the best classification effect. To clearly and intuitively compare the performance of the four classification models as shown in Figures 9 and 10, shown are the ROC curves of the four classification models, and the comparison shows that the deep forest Gcforest algorithm has the best performance [20]. This is due to the high dimensionality of the DNA methylation sequencing data using biomedical sensors in this study, and the multi-granularity scanning structure in the Gcforest algorithm uses a sliding window to preprocess the input data features, and its representation learning ability is further improved. Secondly, the obtained features are input into the cascaded forest of the Gcforest algorithm for training. The cascaded forest combines the input features with the original features. Through the learning of random forests and complete random forests in two-level cascaded forests, compared with logistic regression, Random Forest, Deep Belief Network, and the correlation between features can be learned more fully, so the best performance is obtained. In addition, compared with the deep belief network, the Gcforest algorithm has fewer model parameters and is easy to train, which is more advantageous in small datasets in cancer classification research [21].

RETRACTED

In addition, in this study, a comparative analysis of the influence of different neighbor's *k* and sampling ratio *N* on the comprehensive evaluation index *F*_1_ in the Gcforest classification model is also carried out, the best performance is when *k* = 5.  Table 4 shows the influence of different neighbor *k* and sampling ratio *N* on *F*_1_.

There are two main reasons for the analysis:

1. When the sampling ratio is *N* = 100, the balanced positive and negative sample data still have a large imbalance, which makes the experimental results insignificant.
2. When the sampling ratio is *N* = 300, the number of samples expanded after balancing is much larger than the original samples. Since various oversampling operations such as the SMOTE algorithm are essentially “out of nothing,” the performance of the model after balancing is not obvious as demonstrated in Figure 11. The statement implies a comparative analysis of the influence of different neighbor's *k* and sampling ratio *N* on the comprehensive evaluation index *F*_1_ in the Gcforest classification model. However, in the main study, to address the issue of class imbalance and high dimensionality in The Cancer Genome Atlas (TCGA) massive data, a mixed-sampling imbalanced data ensemble classification technique based on the Intelligent Synthetic Minority Oversampling (SMOTE) algorithm with the aid of biomedical sensors is developed and is essentially a significant model. This leads to a significant increase in the false-negative rate and is used to expand the minority sample set, which effectively improves the classification accuracy of cancer minority class samples under the assumption that the majority class classification accuracy will be maintained.
3. Regarding the selection of the nearest neighbor *k*, when *k* = 3, the model complexity is high, overfitting is easy to occur, and the learning estimation error increases; when *k* = 7, although the learning error is reduced, due to the sample the data set is small, and when *k* is 7, the data far from the sample will also affect the classification result of the model, increasing the approximation error of the model learning.

RETRACTED

## 4. Conclusion

It can be difficult to extract relevant information from the vast amount of healthcare data that wearable computing devices collect and to accurately analyse that data to make an effective diagnosis. To successfully analyse the data that has been taken from biomedical data and analyse it to uncover unrecognized chronic disease signs and forecast a patient's care, artificial intelligence systems and semantic knowledge are required. Additionally, for intelligent healthcare, multitasking deep learning models like Deep Forest that can analyse sensor data are required. This research proposes an integrated intelligent classification model for cancer diagnosis that is embedded with biomedical sensors and uses mixed sampling to overcome the aforementioned problems with the unbalanced data set. The minority sample set is expanded using the intelligent SMOTE technique, and the boundary and noise data are removed using the Tomek Link algorithm. The training data is utilized to significantly increase the classification accuracy of cancer minority class samples after being imported into the Gcforest model, assuming that the classification accuracy for the majority class will be preserved. The experimental findings show that the imbalanced data ensemble classification model embedded with biomedical sensors based on mixed sampling proposed in this paper can significantly increase the classification accuracy of the majority class. This is based on the comparison of models such as Logistic Regression, Random Forest, and Deep Belief Network DBN sensitivity to class. Additionally, when applied to small, unbalanced datasets, the Gcforest classification model using the intelligent SWORT algorithm outperforms the deep belief network DBN. As a result, it tracks real-time data (heart rate, blood sugar, plasma levels, etc.) to assist healthcare professionals in cancer detection. In the future, we hope to employ the suggested framework in conjunction with other cutting-edge machine learning procedures and extraction methods to allow more thorough comparative analyses.

## Figures and Tables

**Figure 1:** The technical flow chart of the research in this paper.

**Figure 2:** DNA methylation data.

**Figure 3:** Cascading forest structure diagram.

**Figure 4:** Decision making process for each forest.

**Figure 5:** Distribution before sampling.

**Figure 6:** Performance indicators of the four models.

**Figure 7:** Distribution sampling.

**Figure 8:** Performance indicators of the four models after mixed sampling.

**Figure 9:** ROC curves of four classification models.

RETRACTED

**Figure 10:** ROC curve graph top left detailed view.

**Figure 11:** Influence of different neighbor *k* and sampling ratio *N* on *F*_1_.

**Table 1:** DNA methylation data used in this paper.

Tumor type	Abbreviation	#patients	Tumor-1	Normal-0
Breast invasive carcinoma	BRCA	885	790	95
Lung adenocarcinoma	LUAD	490	463	34
Urothelial bladder carcinoma	BLCA	435	410	22
Prostate adenocarcinoma	PRAD	546	497	53
Lung squamous cell carcinoma	LUSC	416	370	44
Thyroid cancer	THCA	562	504	59

**Table 2:** Performance indicators of the four models before mixed sampling.

Method	Sen/Rec		Pre		*F*_1_	
	0	1	0	1	0	1
LR	0.705	0.974	0.790	0.976	0.750	0.977
RF	0.795	0.989	0.845	0.990	0.824	0.989
DBN	0.757	0.980	0.825	0.984	0.795	0.977
GcForest	0.834	0.989	0.846	0.994	0.843	0.991

**Table 3:** Performance indicators of the four models after mixed sampling.

Method	Sen/Rec		Pre		*F*_1_	
	0	1	0	1	0	1
LR	0.863	0.980	0.871	0.983	0.868	0.980
RF	0.915	0.989	0.915	0.993	0.919	0.990
DBN	0.895	0.985	0.901	0.987	0.903	0.981
gcForest	0.939	0.987	0.940	0.994	0.936	0.993

**Table 4:** Influence of different neighbor *k* and sampling ratio *N* on *F*_1_.

Experimentalprogram	*N* = 100		*N* = 200		*N* = 300	
	0	1	0	1	0	1
*k* = 3	0.894	0.980	0.914	0.988	0.885	0.981
*k* = 5	0.906	0.990	0.937	0.992	0.894	0.986
*k* = 7	0.887	0.982	0.896	0.988	0.884	0.980

## Data Availability

The data shall be made available on request.
